The article "Simulation Analysis and Study of Gait Stability Related to Motion Joints" was retracted in 2023. Reasons: signs of a paper mill; compromised peer review; unreliable results or conclusions.

# Simulation Analysis and Study of Gait Stability Related to Motion Joints

**DOI:** 10.1155/2022/8417089

**Published:** 2022-07-29

**Authors:** Yuanyuan Lei, Fang Yang

**Affiliations:** Guangxi University of Finance and Economics, Nanning 530007, China

## Abstract

Gait stability in exercise is an inevitable and vexing problem in mechanics, artificial intelligence, sports, and rehabilitation medicine research. With the rapid development and popularization of science and technology, it becomes a reality for researchers to obtain large-scale human motion data sets in real time with higher efficiency. However, at present, the analysis of gait stability of moving joints is still based on image recognition technology, which is ten times less accurate and inefficient. In this paper, Vicon 3D motion capture system, dynamometer, and surface electromyography system were used to obtain the parameters of the lower limbs of the subjects. Using Anywhere modeling and simulation system, simulation experiments were carried out, and the reaction force data of lower limb joints under two environments were obtained. The gait characteristics of human gait were analyzed from the angle of internal and external adjustment mechanism. Combining one-way ANOVA and incremental occupancy rate, the adjustment process of gait stability is described comprehensively. The findings of this study can provide a theoretical basis for the research of lower limb con-assistive devices and can guide the design and development of bipedal anthropomorphic robots.

## 1. Introduction

The average walking movement of the human body in daily life is one of the most basic and main forms of human body movement. In order to meet the needs of the changing living environment, human beings have evolved over a long time to form the body shape and movement system that is most suitable for themselves and the environment, which is also an essential reference for studying human movement and humanoid robots. Therefore, in the simulation of human gait, it is necessary to pay attention to the change of environmental model and movement mode. Kinematics and dynamics analysis of limb and joint movements during walking is very important for analyzing and studying biomechanical factors of lower limbs during stable gait.

Healthy people with normal limb function can keep dynamic balance when walking in normal walking environment under their own neuromodulation system and musculoskeletal movements. However, when a person is influenced by internal factors (such as deformity of lower limbs, insufficient muscle strength of lower limbs, sensory dysfunction, and nerve disorders) or external factors (road obstacles, insufficient ground friction, environmental disturbances, etc.), the person will experience instability during the process of walking. Unstable gait is a common phenomenon in our daily life, which can be caused by slight interference in our body or environment. Among them, fall is a widespread gait instability phenomenon in life, which refers to the human walking process. The center of mass (COM) occurs in the sudden emergency change. Walking individuals cannot rely on their ability to readjust and restore the body balance posture and the phenomenon of slipping and even falling [1]. The slip phenomenon has become an increasingly concerned issue in today's society, especially in the elderly. According to the survey, about 14.7% of the elderly in China fall accidentally every year [2]. According to the survey data released by the World Health Organization. The incidence of falls in the elderly over 80 years of age is 50.0% and the proportion of indoor fall accidents 69.7%. 56.3% of the elderly with a history of falls reported that they had injuries after the fall. It has important social benefits to study the mechanism of gait stability, explore the key factors of gait stability, and restore and compensate the normal activity of people with limb defects to the greatest extent.

The article "Simulation Analysis and Study of Gait Stability Related to Motion Joints" was retracted in 2023. Reasons: signs of a paper mill; compromised peer review; unreliable results or conclusions.

There are many methods to study and analyze human gaits, such as the early traditional footprint method, fixed-point plane camera technology, and 3D analysis system using various sensor technologies. With the popularity of computer technology, virtual technology has been widely applied in various disciplines in recent years. In the computerized virtual environment, human motion modeling and simulation based on human musculoskeletal model systems such as Opensim and Anywhere are gradually applied in the field of gait analysis. This technology makes the gait analysis methods and ideas more diversified and further studies the biomechanics of human body.

In summary, the study of human gait stability is essential for improving people's quality of life and enhancing their sense of well-being. Judging whether the elderly are walking normally by the gait of the human body is of great significance for the elderly to prevent slipping and falling. It has theoretical support in the field of slip and fall prevention. At the same time, it provides a theoretical basis for medical diagnosis, rehabilitation training, and gait planning for anthropomorphic machines such as lower limb walkers, biped robots, and lower limb exoskeletons when walking horizontally and also provides an application reference for walking stability of walking aids such as lower limb exoskeletons.

## 2. Related Work

### 2.1. Gait Stability Study

In the study of human gait stability, scholars at home and abroad have used various methods from different perspectives in different fields to conduct research and discussions in recent years. The causes of gait instability are divided into two main categories: internal factors and external factors. Internal factors mainly refer to individual differences in the human musculoskeletal system, neural control system, and sensory information acquisition and processing ability; external factors mainly refer to environmental differences in ground medium disturbance, shoe sole material texture, and walking environment (such as asynchronous path environment, gravity environment, visual environment, and auditory environment) [3]. The following section will review the status of research in gait stability concerning the above two factors.

The article "Simulation Analysis and Study of Gait Stability Related to Motion Joints" was retracted in 2023. Reasons: signs of a paper mill; compromised peer review; unreliable results or conclusions.

In terms of internal factors studies, Hamacher et al. showed that by studying gait stability, characteristics of 10 young and 18 older adults walking after physical exhaustion that older adults walking at maximum fatigue are less stable and may exhibit a higher risk of falling and predict and prevent falls by walking gait in fatigue state [4]. Terrier and Reynard tested the gait characteristics of 8 children with developmental coordination disorder and 10 normally developing children walking on a treadmill for 4 minutes and concluded that children with developmental coordination disorders can be detected by their local dynamic stability while walking. The effect of age on gait stability was analyzed through experiments on 100 healthy subjects aged 20-69 years and showed a significant association between age and gait instability; in addition, gait instability may start to increase at a faster rate at the age of 40-50 years [5]. Simon et al. assessed dynamic gait imbalances in patients with spinal deformities by conducting a comparative study of gait in 12 normal subjects and 17 patients with spinal deformities and showed that patients with column misalignment exhibited reduced gait stability, symmetry, and consistency [6]. Kurz et al. investigated whether injurious stimuli (hypertonic saline injections) in the low back or calf muscles affected gait stability. The results showed that the effect on gait stability depended on pain location and walking speed, which showed that back pain had a more significant effect on gait stability than calf pain [7]. By comparing the gait characteristics of children with cerebral palsy with those of healthy developing children, Kurz et al. found that children with cerebral palsy had poor gait stability because they needed more stride length to eliminate the disturbances present [8].

The article "Simulation Analysis and Study of Gait Stability Related to Motion Joints" was retracted in 2023. Reasons: signs of a paper mill; compromised peer review; unreliable results or conclusions.

In the study of external factors, Daniel H et al. studied 25 healthy elderly subjects in two auditory environments, regular and active noise cancellation, to analyze local dynamic gait stability and showed the improvement in gait stability of subjects during regular ground walking when active noise cancellation was used compared to normal hearing. Hyunsoo K et al. studied five experienced steel erectors and 11 inexperienced workers walking on smooth-coated steel frames in gait stability; the results of this study highlight the use of gait stability to quantitatively predict the safety risk posed by smooth-coated steel beams. For M et al. who measured the effect of dual tasking on gait stability in 15 healthy male young adults walking on different inclined steps, the results showed that reducing gait speed under dual tasking was an essential factor in improving dynamic stability and optimize performance on the secondary task as compensation and that changes in walking speed and center of the mass position may be vital in avoiding hazards and preventing falls and increasing dynamic gait stability. By studying gait index changes and gait stability characteristics in 19 young men during the same walking task in different environments (indoor and outdoor), Paola T et al. showed that both environmental and test conditions affect gait change indices for young, healthy adults but not gait stability indices. Xing YC et al. investigated the effect of backpack loading on stair gait in young male adults. They showed that subjects adjusted their postural control to compensate for disturbances due to backpack loading and maintained their postural stability in the unloaded state but may experience an increased risk of stair contact during uphill increased and an increased risk of overstepping during stair descent.

### 2.2. Human Body Mechanics Model Construction and Simulation Analysis

The structure of human lower extremity is very complex, and the force of each joint and muscle especially during walking is difficult to measure directly. The construction of lower extremity mechanics model by analyzing the force during walking can provide the basis for the analysis of human walking mechanism and the development of lower extremity rehabilitation aids and lower extremity exoskeletal devices. There are many software programs for human motion and dynamics simulation through musculoskeletal modeling, such as OpenSim, LifeMOD, and AnyBody. Therefore, it is important to study the mechanics model construction through computerized musculoskeletal modeling of human lower limbs. In this paper, the computer model and Vicon 3D motion capture system are used to simulate human gait.

The article "Simulation Analysis and Study of Gait Stability Related to Motion Joints" was retracted in 2023. Reasons: signs of a paper mill; compromised peer review; unreliable results or conclusions.

As far as foreign studies are concerned, Yeadon established a multirigid body mechanics model in 1964, consisting of 15 multirigid links connected by a spherical hinge system [9]. Hurwitz et al. analyzed the stresses on lower limb joints during human motion by constructing a static mechanical model of the human lower limb [10]. Damsgaard et al. constructed a musculoskeletal system by analyzing the skeletal structure characteristics of humans and other organisms and solved the inverse dynamic problem of the basic uncertainty of muscle structure [11]. Alexander and Schwameder analyzed the load differences in lower extremity joint compressive force and tibiofemoral joint shear force during inclined walking at different inclinations [12]. Petrone et al. used OpenSim and the AnyBody system code to analyze the isokinetic. The musculoskeletal model was validated experimentally during knee flexion and extension [13]. Michalina et al. used the musculoskeletal model in the OpenSim software system to determine ankle joint muscle force magnitude changes during gait. Tito B et al. imported motion data into AnyBody to set up the model kinematics and calculated intersegmental loads at the L4L5 level during each task. The calculated loads were processed according to two different methods to obtain the corresponding intradiscal pressures compared with the in vivo measurements. The results were also compared with the measurements to assess the accuracy of the lumbar pelvic kinematics. Bruijn and Van explored the usability of the AnyBody modeling system based on a skeletal muscle model in assessing the ability to apply forces at different points in the workspace and various directions of motion [14]. It can be found that although many scholars have analyzed the mechanical structure model of human body, their research is more aimed at medical health inspection, and there is not much simulation analysis of mechanics.

## 3. Gait Analysis and Stability Study of Human Sports Joints

### 3.1. Gait Biomechanical Parameters

#### 3.1.1. Gait Cycle

Completing human walking action needs to meet two conditions: (1) each foot from a support point to the next support point for periodic movement and (2) the ground support force is sufficient to support the body movement. The mechanical characteristics of these two conditions can be detected and simulated by computer. Human gait is a periodic movement; a complete gait cycle is defined as a walking process, from any side of the heel touching the ground as the beginning to the same side of the heel touching the ground again as the end of this period. The whole gait cycle can be divided into two phases: the support phase and the swing phase, in which the support phase accounts for about 60%-62% of the whole gait cycle and the swing phase accounts for about 38%-40% of the whole gait cycle, further subdivided into four phases, including the first double support phase, the single support phase, the second double support phase, and the swing phase, where we take the first step. The right foot is used as an example to make a brief clarification.

1. The first double support phase: the right foot heel touching the ground as the beginning and the left foot toes off the ground as the end, accounting for about 10%~12% of the gait cycle. At this stage, the body's center of gravity is gradually shifted to the right foot entire foot
2. Single support phase: beginning with the left foot toes off the ground and ending with the left foot heel touching the ground, accounting for about 38%~40% of the gait cycle. In this phase, the left foot is used as the swing leg to complete the striding action, and the right foot is used as the supporting leg to bear all the gravity of the body
3. The second double support phase: the left heel touches the ground as the beginning, and the right toe leaves the ground as the end, accounting for about 10%~12% of the gait cycle. At this stage, the body's center of gravity is gradually shifted to the left foot's entire foot due to the preparation of the stirrup action afterward
4. Swing phase: the swing phase starts with the toes of the right foot leaving the ground and ends with the heel of the right foot touching the ground again, accounting for about 38%~40% of the gait cycle. In this phase, the right foot is used as the swing leg to complete the striding action, and the left foot is used as the supporting leg to bear all the gravity of the body

The article "Simulation Analysis and Study of Gait Stability Related to Motion Joints" was retracted in 2023. Reasons: signs of a paper mill; compromised peer review; unreliable results or conclusions.

#### 3.1.2. Time and Space Parameters

Time parameters mainly include gait speed, gait frequency, gait cycle, support phase time, and swing phase time. Gait speed usually refers to the walking unit of time in the direction of travel displacement called step speed, usually expressed in m/s; healthy people usually walk at a speed of about 1.0-1.6 m/s. Gait frequency refers to the number of steps per minute called step frequency or pace; healthy people usually gait frequency is about 95-125 steps/min, fast walking up to 140 steps/min. Stride time refers to the time taken to complete a gait cycle. The setting of time parameters is based on the previous studies and internationally recognized speed and frequency, so the identification in this paper is limited to ordinary people.

Spatial parameters mainly include stride length, stride width, stride width, and foot angle. The stride length is the longitudinal distance between the left and right heel (or toe) when walking in a straight line. According to the data from official websites such as China Bureau of Statistics and Health Bureau, it can be determined that the stride length of young Chinese men is about 55.0-77.5 cm, while the stride length of young women is about 50.0-70.0 cm. Stride width also called the base of support (BOS) refers to the lateral distance between the center points of the heels or gravity points on both sides of a step. Foot angle refers to the angle formed by the centerline through the sole of one foot and the forward direction, which characterizes the degree of internal and external rotation of the lower limb when standing, as shown in Figure 1.

The article "Simulation Analysis and Study of Gait Stability Related to Motion Joints" was retracted in 2023. Reasons: signs of a paper mill; compromised peer review; unreliable results or conclusions.

#### 3.1.3. Kinematic Parameters

Kinematics is a branch of mechanics that describes and studies the changing law of an object's position with time from a geometric point of view (referring to the physical properties of the object itself and the force exerted on the object). Kinematic parameters are used to describe the movement of the human body in space. They are a reflection of the laws of hip, knee, and ankle joint movement (angular change or displacement, velocity, acceleration, etc.), the laws of change in the position of the body's center of gravity, and the laws of change in the position of the pelvis. According to the anatomical theory, when the human body walks, the movement mainly occurs on three surfaces: the sagittal plane, coronal plane (frontal plane), and horizontal plane (transverse plane). This is shown in Figure 2. Sagittal plane: the plane through the vertical uranium and longitudinal axis and all the planes parallel to it are called the sagittal plane. The median sagittal plane divides the body into two symmetrical parts, left and right. Coronal plane: the plane through the vertical and horizontal axes and all the planes parallel to it are called coronal planes. The median coronal plane divides the body into two symmetrical parts, front and back. Horizontal plane: all the planes perpendicular to the sagittal plane and coronal plane are called horizontal planes. The median horizontal plane divides the body into two symmetrical parts: upper and lower.

### 3.2. Gait Stability

The focus of this study is to outline the internal and external factors affecting gait stability during human walking; human stability is the ability of the human body to effectively transfer energy and maintain the balance of body posture in the trunk position at rest or in motion; stability is also known as the degree of stability or stability. The stability of the human body is divided into two cases: one refers to the ability of the human body at rest to resist various external disturbances, known as static stability; the second refers to the body's center of gravity shift balance position; the body can still maintain a balanced movement when disturbed by external factors, known as the dynamic stability of human balance. The gait stability studied in this paper is the second case of dynamic stability.

The article "Simulation Analysis and Study of Gait Stability Related to Motion Joints" was retracted in 2023. Reasons: signs of a paper mill; compromised peer review; unreliable results or conclusions.

#### 3.2.1. Factors Influencing Gait Stability

The human body maintains a finite stable equilibrium under support to evaluate the stability of whether it is easy to lose balance, easy to lose balance is weak stability, and not easy to lose balance is strong stability, which are the factors affecting stability. In this paper, taking the internal and external factors that affect the balance of human body as reference, in order to facilitate calculation, mechanical factors and biological factors are set.

*(1) Mechanical Factors Affecting the Balance of the Human Body*.

1. The height of the center of gravity of the human body affects human balance; the higher the position of the center of gravity, the weaker the stability; the lower the position of the center of gravity, the stronger the stability. For example, when the human body is sliding downhill, the center of gravity needs to be lowered to keep the body stable; in handstand exercises, when there is a risk of losing balance, this can be adjusted by bending the elbows to lower the center of gravity
2. The size of the support surface (BOS) affects the human body balance; the so-called support surface is the area enclosed by the edge of the support point, for example, the support surface when standing bipedal, as shown in Figure 3. The larger the support surface, the stronger the stability; the smaller the support surface, the weaker the stability. For example, standing on both feet is more stable than standing on one foot, and walking on a tightrope is more complex than walking on a balance beam
3. The size of the stability coefficient affects the stability of the human body; if in the human body balance, there is interference from external forces, then there is a balance of the human body and the ratio of the stabilizing moment and the overturning moment; their ratio is called the stability coefficient *K*. If *K* > 1, the human body can resist the external overturning moment to maintain stability; if *K* < 1, the human body cannot resist the external overturning moment, and the human body balance is damaged to produce instability phenomenon
4. The size of the body mass also affects the stability of the human gait; the larger the body mass, the stronger the stability; the smaller the body mass, the weaker the stability. This is also the reason why in wrestling matches, the weight is graded according to the competition
5. The static friction between the foot and the ground also affects the stability of the human body. Obviously, the greater the friction, the stronger the stability; friction is small, the weaker the stability

*(2) Biological Factors Affecting the Balance of the Human Body*. The human body cannot be static due to the influence of respiration and blood flow in the human body, resulting in subtle dynamic changes in the body's center of gravity. At the same time, the tension of the whole body muscle groups cannot be constant at any time and always produces deviations from the counterforce, so the human body does not exist absolute rest.

The article "Simulation Analysis and Study of Gait Stability Related to Motion Joints" was retracted in 2023. Reasons: signs of a paper mill; compromised peer review; unreliable results or conclusions.

The effective support surface for human balance is smaller than the actual support surface, because the human body is not a static shape. The human body is often unable to maintain balance due to insufficient soft tissue and muscle strength, so when gravity acts on the edge of the supporting surface, a tipping situation occurs. When the body tends to topple over, it will reflexively change the body posture, generally the total center of gravity of the body, to the opposite direction of displacement (called compensatory action or compensatory movement).

The human body has a certain ability to adjust balance. When the human body cannot reach a balanced position or is in danger of losing balance, it can be adjusted through visual and physical sensations (muscle receptors and vestibular apparatus) under the control of the cerebral cortex, thereby causing corresponding muscle tension and contraction. This instinct of the human body to maintain and restore balance can be highly automated through later training.

Human balance is affected by psychological factors; in the process of human walking, changes in the external environment and changes in the human body's internal environment will have a certain impact on the human nervous system, which is expressed in the change of psychological factors. Among them, the psychological reaction of tension has the most obvious impact on the stability of the human body. On the one hand, tension will affect the regulatory role of vision in balance regulation; on the other hand, it will also affect the ability of the brain and the nervous system to regulate the body's muscles. The human body balance action consumes the physiological capacity of the muscles; in the walking process, the size of muscle strength is an important factor affecting stability. The muscles of the body link to make the corresponding restraint work, through the link of the muscle pull moment, increase the external moment of support restraint to offset the external resistance moment and the body link of the heavy moment to maintain a certain balance posture.

The article "Simulation Analysis and Study of Gait Stability Related to Motion Joints" was retracted in 2023. Reasons: signs of a paper mill; compromised peer review; unreliable results or conclusions.

#### 3.2.2. State Stability Evaluation Method

In order to evaluate the level of stability of the human body in nonfall situations, various mathematical methods for evaluating stability have gradually been developed. At present, the main analyses of gait stability are comparative studies of normal and abnormal groups, comparative studies of influencing factors, comparative studies of different age groups, etc., and all these studies have the necessity of quantitative analysis of stability.

*(1) The Center of Mass Projection Analysis Method*. In the early days of gait stability research, most researchers believed that the body's center of gravity was one of the important factors affecting gait stability. The relationship between the center of mass (COM) or center of gravity (COG) of the body and its support surface (BOS) was used to determine the stability of the individual. However, the human body is not static stability during walking, but dynamic stability that constantly changes the stability state. Only the relationship between the body's center of mass and the support surface is considered insufficient to evaluate stability. When the body completes the sit-up-walking action, from the sitting position to the standing state, the center of mass is projected outside the support surface. According to the static center-of-mass projection method, the body should be unstable and may fall. However, under normal circumstances, the body can be carried out through its adjustment mechanism to the standing state and will not fall. For this phenomenon, some correction methods are proposed, such as the dynamic mapping relationship of the center of mass concerning the support surface.

*(2) Traditional Data Variability Methods*. The traditional parameters for evaluating stability by kinematic data are step length, step width, walking duration per walking cycle, displacement of the center of gravity position during walking, etc. A common method to evaluate these parameters is to calculate their standard deviation and coefficient of variation. Because these methods have the meaning of how discrete the data points are about the overall mean of the data, they represent the degree of variability of the data. The coefficient of variation (CV) is a statistical measure of the degree of variation of the observations in the data. The coefficient of variation, like the extreme deviation, standard deviation, and variance, is an absolute value that reflects the degree of dispersion of the data.

*(3) Nonlinear Time Series Analysis Method*. The human body is a nonlinear multisystem, the system is in dynamic equilibrium for a long time, and with the continuation of time, the cycle of steady state to an unstable state to new stable state is constantly repeated. At the same time, variability also exists all the time, and it is due to the existence of variability that the original state of the system is changed to another state, thus forming a nonlinear dynamic system. The nonlinear time series analysis method examines the relationship between sampled data and time. Analyzing the variability of biorhythmic signal fluctuations in the human body requires a deeper exploration of spatiotemporal parameters. The research method used in this paper is a reference to this approach to investigate the characteristics of dynamic variability of individual parameters over time. In this paper, the nonlinear time series analysis method is selected as a reference, and some cases are improved, which makes the algorithm more suitable for Chinese physique.

The article "Simulation Analysis and Study of Gait Stability Related to Motion Joints" was retracted in 2023. Reasons: signs of a paper mill; compromised peer review; unreliable results or conclusions.

## 4. Gait Stability Simulation Experiment and Analysis

### 4.1. Human Model Simulation System

AnyBody is a musculoskeletal modeling system for biomechanical simulations to analyze the human body's reactions in vivo or between the body and the environment. This includes things that are implanted inside the body (implants, knee or hip devices, etc.), external attachments (exoskeletons, knee pads or space suits, etc.), or things that interact with the body (car seats, wheelchairs, etc.), as shown in Figure 4.

AnyBody system has a diversity of inputs and outputs. AnyBody uses motion as input, which can be done using the most common motion capture (MoCap) system, Vicon, but can also handle MoCap data (C3D format) from many other systems. Also, in AnyBody, it is possible to define your motion by manually defining the initial joint angle and joint velocity. The results are output by inverse dynamics analysis, kinematic analysis, or optimization analysis, including data such as muscle activation or not, joint reaction force, joint moment, and user-defined types, and the output file formats include pictures, graphs, and text.

There are two main types of models in the human musculoskeletal system model: forward kinetics model and inverse kinetics model. Forward dynamics is based on the assumption of muscle activity to calculate the kinematic parameters of the model. This model is very suitable for specific simulations of various physical phenomena and is a computationally intensive optimal control problem that requires much optimization to drive the model to accomplish a specific task. AnyBody allows only inverse dynamics analysis of the model, and its solution to the muscle problem can be summarized as an optimization problem of the following form.

(1) $$\begin{array}{c} \left\{\begin{array}{c} MinG\left(f^{\left(M\right)}\right)\\ \text{Subject }toCf^{\left(M\right)}=d\\ 0\leq f_{i}^{\left(M\right)}\leq N_{i},i\in \left\{1,2,\cdots ,n^{M}\right\}, \end{array}\right.\\ G\left(f^{\left(M\right)}\right)=\text{Max}\left(A_{i}^{M}\right)=\text{Max}\left(\frac{f_{i}^{\left(M\right)}}{N_{i}}\right), \end{array}$$

where *G* is the objective function, i.e., the standard selected strategy for the assumed central nervous system; *f*^(*M*)^ is the muscle force; *N*_*i*_ is the muscle strength, i.e., the maximum force that the muscle can provide at its optimal length; *a*_*i*_^*M*^ is the muscle mobility, i.e., the ratio of muscle force to its strength; *C* is the system coefficient matrix; *d* is the external force applied to the human system, in this study, the ground support reaction force; and *n*^*M*^ is the number of muscles in the model.

The article "Simulation Analysis and Study of Gait Stability Related to Motion Joints" was retracted in 2023. Reasons: signs of a paper mill; compromised peer review; unreliable results or conclusions.

### 4.2. Motor Joint Human Lower Limb Musculoskeletal Model Construction

The AnyBody model simulation system used for the simulation analysis in this study is Version 6.0.1. In this paper, the application model “MoCapModel” provided in the model library of AnyBody model simulation system is used as the basis. The application is modified according to the actual situation of the experiment, and the specific steps are as follows.

1. The computational load of the AnyBody software for the inverse dynamics analysis of human motion is huge and time-consuming, so the C3D files obtained in all experiments are subjected to gait cycle interception to reduce the redundant computations during the software computation. Therefore, the experimental data for the 13 subjects on dry and slippery roads were examined and screened and preprocessed 10 times each to prepare for importing the data
2. Open AMMR-Application-Examples-MoCapModel-MoCap-FullBody.main and press F7 to load the model, and open the ModelView window to observe the model in real time. The content of this study is human lower extremity movement, so the upper extremity of the model should be constrained in the system; change the value 1 of Use Upper Extremities in the main program to 0, and load the model
3. After completing the above adjustments, first build the skeletal model for kinematic simulation analysis; this process does not require the participation of muscle parts; change the Motion And Parameter Optimization Model from 0 to 1 in the AnyBody main program, and change the Inverse Dynamic Model from 1 to 0, and load the model
4. At this time, load the experimental data C3D file; here, zhidaowu01.c3d file is an example. Import the C3D file into the AMMR-Application-Examples-MoCapModel-Input folder and open the TrialSpecificData.any file that will replace the import file name zhidaowu01.c3d, and load the model. When an error is generated, go to the next operation
5. Since the subjects and the experimental environment of this experiment are different from the existing models in the model library, they should be modified according to the actual situation. First of all, as far as the experimental environment is concerned, this experiment uses 4 force tables. At the same time, there are only 3 in the model, so open Environment-any-ForcePlants.any in the program to make changes and calibrate the force plate type for the force tables. Secondly, for the experimental subjects, the size of the manikin in the actual experimental data is different from the size of the existing model, so the parameters of the manikin are modified to the basic information parameters of the subjects and loaded into the model
6. Due to the irresistible error in the experiment, after importing the subject's C3D file, there is a difference between the actual blue marker points collected by the subject and the red marker points of the model itself, so the coordinates of the blue points in *X*, *Y*, and *Z* directions are adjusted to make them infinitely close to the red points, and the best result is that they overlap completely, as shown in Figure 5
7. After completing the above adjustments, the kinematic analysis of the human lower limb skeletal model can be performed as Operations—Motion Optimization—Initial Conditions—Kinematics program, specifically. The process of kinematic simulation analysis is shown in Figures 6 and 7
8. After the kinematic analysis, reverse dynamics analysis should be performed. Change Motion And Parameter Optimization Model from 1 to 0 and Inverse Dynamic Model from 0 to 1 in AnyBody main program, and load the model. Run the Operations—Motion Optimization—Initial Conditions—Inverse Dynamics program, and the process of inverse dynamics analysis is as follows. The process of inverse dynamics analysis is shown in the figure below. In the process of the inverse dynamics simulation, the force of the lower limb muscles will change with the change of the human gait movement. The reflection on the human musculoskeletal model is the color change of the corresponding muscles; the greater the force, the darker the color of the muscles will be. The initial state of the muscle color is light. The blue line in the figure indicates that the force table measured the ground on the body's support and reaction force and real-time dynamic changes

The article "Simulation Analysis and Study of Gait Stability Related to Motion Joints" was retracted in 2023. Reasons: signs of a paper mill; compromised peer review; unreliable results or conclusions.

### 4.3. Kinematic Joint Human Lower Limb Musculoskeletal Model Validation

After building a human musculoskeletal model in the AnyBody system, the model needs to be validated to ensure the accuracy of the constructed human musculoskeletal model and the validity of the simulation parameters. Using a method proposed by Dkkerson et al. that compares the simulated muscle forces with the subject's EMG parameters, this method allows for semiquantitative validation of the simulation model's ability to calculate muscle forces. In order to perform a progressive semiquantitative validation of the lower limb musculoskeletal model, the two were tested using the Pearson correlation coefficient, also known as the product-moment correlation coefficient, which is a statistical indicator capable of quantitatively describing how good the linear correlation is, and the analysis is shown in Table 1.

The correlation analysis shows that the correlation coefficients of the four muscles are higher than 0.5. It can be proved that the surface EMG signals and simulated muscle forces of the four muscles, biceps femoris, semitendinosus, tibialis anterior, and lateral gastrocnemius are significantly correlated, and the same model is used for the same subjects in the oiled ground environment and the dry ground environment, and the validation results are not repeated. In summary, the validity of the human musculoskeletal model in the AnyBody system can be demonstrated, and the results simulated by this model can be used for further analysis and research.

### 4.4. Simulation Experiment Analysis

Through the inverse dynamics simulation analysis of AnyBody system, the parameters of joint contact force changes of hip, knee, and ankle joints during human lower limb walking can be obtained. The internal factors of joint reaction forces during human lower limb walking will be analyzed.

Joint reaction forces, also known as contact forces at the joints, are divided into three main types: near and far forces, anterior and posterior forces, and internal and external forces, and this section will analyze the joint reaction force changes from three joints of the lower limb movement.

As shown in Figure 8(a), the hip joint distal and proximal reaction forces were mainly manifested as the distal force. The bimodal characteristics appeared in both the dry and oiled environments. However, the first peak value of the hip joint distal force in the oiled environment was significantly smaller than that in the 1,000-dry environment, and the second peak was slightly smaller than that in the dry environment. As shown in Figure 8(b), the hip joint front and rear reaction force changes in a similar trend, but in the first double support phase and single support phase (i.e., before the 40% gait cycle), the forward walking force in the oiled environment is greater than that in the dry environment and in the second double support phase and support phase before the dry environment is smaller than that in the dry environment, which is due to the body center of gravity swaying under the disturbance of the oil medium, and the hip joint maintains the body by adjusting the front and rear end force balance. As shown in Figure 8(c), the trend of force reflected inside and outside the hip joint was the same, and the hip joint had a lag in the inward end force when disturbed by the oil medium and then recovered the same as the dry environment.

The article "Simulation Analysis and Study of Gait Stability Related to Motion Joints" was retracted in 2023. Reasons: signs of a paper mill; compromised peer review; unreliable results or conclusions.

As shown in Figure 9, the knee joint reaction force walking in the dry environment all exhibited obvious bimodal characteristics. However, in the oiled environment, the first peak value phenomenon was significantly weakened. Within the first double support phase, the knee joint mainly exhibited distal, posterior, and outward forces. The knee joint distal, posterior, and outward forces during walking in the oiled environment were smaller than those in the dry environment. In the single support phase, the absolute values of the distal, posterior, and outward forces were smaller than those in the dry environment in the early phase. However, in the late phase of the single support phase, the distal, posterior, and outward forces of the knee joint in the oiled environment increased rapidly. They were larger than those in the dry environment. In the second double support phase, the knee joint's distal, backward, and outward forces in the oiled environment were consistently greater than those in the dry environment. The two environments in the oscillation phase had the same trend and similar force values. It can be seen that during walking, the knee joint regulates the body balance by weakening the distal, backward, and outward forces during the phase from when the foot first touches the oil surface to when the foot is completely flat while increasing the distal, backward, and outward forces during the later part of the but-support phase, i.e., when the foot leaves the oil surface to move forward, to make the body move forward smoothly.

As shown in Figure 10(a), the ankle joint distal and proximal reaction forces were mainly forward in both environments, similar to the knee joint. The bimodal characteristics weakened in the oiled environment. As shown in Figure 10(b), the anterior and posterior reaction forces of the ankle joint in both environments mainly showed forward force. The changing trend of both was the same. However, the forward force of the ankle joint in the oiled environment was much larger than that in the dry environment, which was due to the fact that the ground could not provide sufficient friction under the oil medium disturbance. The ankle joint maintained the motion by increasing the previous force. As shown in Figure 10(c), the trends of internal and external reaction forces of the ankle joint were similar in the two environments, with the absolute values of outward force in the oiled environment being smaller than those in the dry environment and the absolute values of inward force being larger than those in the dry environment. This is due to the tendency of the foot to slide outward under the perturbation of the oil medium, and the human body, in order to avoid the outward slip to produce a fall, weakens the outward force and enhances the inward force to overcome the slip.

The article "Simulation Analysis and Study of Gait Stability Related to Motion Joints" was retracted in 2023. Reasons: signs of a paper mill; compromised peer review; unreliable results or conclusions.

In summary, comparing the three joints of the hip, knee, and ankle, the hip joint > knee joint > ankle joint in terms of near and far reaction force; ankle joint > knee joint > hip joint in terms of front and back reaction force; and hip joint > knee joint > ankle joint in terms of internal and external reaction force. Under the constant perturbation of oil medium, in the support phase, each joint regulates the walking balance by first reducing the near and far reaction force and the internal and external reaction force and then rapidly increasing them. At the same time, the hip and ankle joints overcome the influence of oil medium perturbation by enhancing the forward reaction force to achieve stable walking.

## 5. Conclusion

In this paper, based on the gait movement data of subjects collected in gait test, the simulation of lower limb movement is carried out by using the Anyhow human body model simulation software, and the variation curves of reaction forces of ankle joint, knee joint, and hip joint are compared and analyzed when the human body walks in the dry land environment and oil land environment.

Firstly, a musculoskeletal model of human lower limbs was constructed in AnyBody model simulation system, and the C3D file obtained in the experiment was used to complete the driving of the model. Inverse dynamics simulation analysis is carried out, and the parameters of joint reaction force changes are obtained. Secondly, by comparing the surface EMG signals and simulated changes of biceps femoris, semitendinosus muscle, tibialis anterior, and lateral gastrocnemius muscle, the lower limb musculoskeletal model was verified, and the Pearson correlation analysis was carried out to verify the validity of the lower limb musculoskeletal model. Finally, the joint reaction forces of lower limbs, hip joints, knee joints, and ankle joints were analyzed. In the aspect of joint reaction force, each joint in the supporting stage adjusts walking balance by reducing distal and proximal reaction force and the internal and external reaction force at first and then increasing them rapidly. At the same time, the hip and ankle joints can overcome the influence of oil disturbance by strengthening the forward reaction force and realize stable walking.

The article "Simulation Analysis and Study of Gait Stability Related to Motion Joints" was retracted in 2023. Reasons: signs of a paper mill; compromised peer review; unreliable results or conclusions.

## Figures and Tables

**Figure 1:** Spatial gait parameters.

**Figure 2:** The planes and axis of human anatomy.

**Figure 3:** Support surface.

**Figure 4:** AnyBody human model simulation system.

**Figure 5:** Kinematic analysis before and after adjustment of marker points.

**Figure 6:** Kinematic simulation analysis chart.

**Figure 7:** Reverse dynamics simulation analysis chart.

**Figure 8:** Hip reaction force.

**Figure 9:** Knee reaction force.

**Figure 10:** Ankle reaction force.

**Table 1:** Correlation coefficient table between muscle force and surface EMG signal.

Muscle name	Tibialis anterior muscle	Semitendinosus	Biceps brachii
Correlation coefficient	0.863	0.873	0.664

## Data Availability

No data were used to support this study.
